# A Systematic Review and Meta-Analysis on Comparative Kinematics in the Lumbopelvic Region in the Patients Suffering from Spinal Pain

**DOI:** 10.1155/2022/7369242

**Published:** 2022-03-19

**Authors:** ZhiRui Zheng, YouQiang Wang, Tong Wang, Yue Wu, YuHui Li

**Affiliations:** The Second Affiliated Hospital of Harbin Medical University Orthopedic Surgery Three Ward, Harbin, Heilonjiang, China

## Abstract

**Background:**

Lumbopelvic kinematics has been observed to include different parameters and directly relate to the movement of the hip spine. In the current scenario, more than 65 million people have been suffering from spinal pain, and 18% of adults experience chronic spinal pain.

**Methods:**

This systematic review and meta-analysis selected 9 studies for analysis via electronic databases like EMBASE, MEDLINE, Web of Science, Scopus, CINAHL, and Cochrane (CENTRAL). After collecting the data, the dataset has been systematically analyzed through statistical methodologies using RevMan and Stata.

**Results:**

Out of 116 studies initially scrutinized, nine were finally selected for the meta-analysis. When range of motion was studied via meta-analysis, it was noted that a considerable reduced movement was noted in the lumbar region of the spine when people were suffering from lower back pain in comparison to control group people. Hence, reduced lumbar range of motion, no difference in the angle of lordosis, and no significant difference in extension and rotation in people with lower back pain were found. However, variability was noted in people suffering from lower back pain for flexion and lateral flexion. A significant heterogeneity was found between the studies which lacked some details and standardization of the criteria which were used for defining patients with lower back pain or without them (control group). Results show that spinal pain is the main reason behind the limitation of lumbar range of motion. It is clear from the data set of mean and standard deviation, and this is clear to establish the relationship between the causes of pelvic and spinal pain. In flexion-based ROM, the mean difference was found to be −9.77 (95% CI: −21.86, 2.32). Similarly, for lateral flexion, the mean difference was found to be −5.58 (with 95% CI: −10.38, −0.79).

**Conclusion:**

It can be concluded that spinal disease is too influential for people; thereby, it affects day-to-day life activities by creating painful and restricted movements. It is concluded that people suffering from lower back pain have reduced proprioception and range of movement in the lumbar region when compared to control groups with no lower back pain, which mainly focus on flexion and lateral flexion.

## 1. Introduction

Lumbopelvic kinematics have been observed to include a wide range of parameters, such as lumbar and pelvic ROM, regional movement timing, and muscle activation. In addition to that, the duration of movement and postural position associated with the coordination of movement are also linked with lumbopelvic kinematics. The lumbopelvic rhythm for the coordination of the hip-spine can be described as the movement of the lumbar spine combined with the movement of the pelvis. The lower back muscle, called the erector spinae, contracts and relaxes to control the body's movement against gravity [1].

It has also been observed that the nerves in the pelvic region come from the lower back portion, and issues with the lumbar spine can contribute to the development of pelvic pain or spine pain. In addition to that, the other potential causes of lower back disorders associated with spine pain can be triggered by disc herniation, spinal stenosis, and pinched nerves [2]. This study will systematically review and provide a meta-analysis on the comparative kinematics in the pelvic region for patients who are suffering from spinal pain. In addition to that, this study will also shed light on the finding of possible solutions to mitigate the issues related to spinal pain [3].

This study aims to systematically review and produce a meta-analysis on the comparative research regarding kinematics in the lumbopelvic region for patients suffering from spinal pain. The key objectives of the study are as follows: (i) to analyze the current scenario of developing lumbopelvic disorders among patients suffering from spinal pain; (ii) to investigate the importance of kinematics in the lumbopelvic region; and (iii) to examine the possible ways of improving strategies to mitigate the issues associated with the lumbopelvic region.

Spinal pain has been observed to be a common disorder among adults from the age group of 40 to above 60. In the current scenario, more than 65 million people have been suffering from spinal pain. At the same time, 18% of adults have been found to experience chronic or persistent spinal pain because of certain daily activities [4].

Therefore, this has become a potential issue nowadays and needs to be controlled. In this regard, this study will systematically review and provide a meta-analysis on the comparative kinematics for the lumbopelvic region among patients suffering from spinal pain. This study will analyze different perspectives of other researchers through conducting a secondary systematic review that can contribute to finding something new in the process of creating this kind of spinal pain. Therefore, this study will also contribute to the development of strategies and procedures that can effectively reduce the number of individuals suffering from spinal pain through conducting a systematic review and meta-analysis.

## 2. Methodology

The methodology can be defined as conducting research, describing each step selected and completed in research. This study has been conducted with a systematic review of secondary sources that has presented a meta-analysis regarding the research topic [5].

### 2.1. Study Selection: Inclusion and Exclusion Criteria

The inclusion-exclusion criteria have been chosen to identify the selected population in this study as a reliable, consistent, uniform, and objective manager. At the same time, the selected source of data has also been passed through these inclusion and exclusion criteria. It has lowered the size of the population by removing the ineligible samples from the study. Databases such as EMBASE, MEDLINE, Web of Science, Scopus, CINAHL, and Cochrane (CENTRAL) were used for data extraction.

A PRISMA flow chart has been implemented to systematically include and exclude studies from this review work and meta-analysis. Records identified through electronic database searching have collected 113 studies from different sources. After that, three additional articles have also been included in this study from other sources.

Out of these 116 studies, 76 duplicate types of research were discarded. Following the inclusion criteria and eligibility standards, 40 studies were found applicable as per the aim of the current study. Articles were rejected as per their exclusion criteria, which were as follows: insufficient patient data, nonclinical studies, studies with no conclusions, review papers, abstracts, letters, or editorials were found to be 31 studies; therefore, nine studies were shortlisted for analysis (Table 1). The PRISMA statement flow chart shows this process (Figure 1).

In this systematic review and meta-analysis study, four major electronic databases have been searched systematically since November 2021. Electronic databases including PubMed, Google Scholar, ProQuest, and MEDLINE have been searched with specific combinations of keywords. The selection of articles from the data sources has been conducted with relieving the abstracts and titles of the journals.

Online data sources have contributed to this research and have helped the researchers conduct these meta-analyses and systematic reviews. During the data search, researchers selected only the journals related to this topic and used a bulletin table to search the most relevant journals [14]. In this secondary data collection, the researchers have also considered the relevance and eligibility of each online source that has been reviewed in this study. During the selection of online sources, the researchers chose different clinical studies, individual participant data, regulatory information, and other types of secondary data that are relevant to the review topic.

### 2.2. Data Extraction and Quality Assessment of the Study

Researchers have developed based on the checklist used in different articles and published the quality assessment tools to extract data from the collected sample. Data extraction and quality assessment have been necessary to reduce risk factors and bias in the systematic review while synthesizing the key findings. The characteristics included in the data extraction were the age of participants and the characteristics of the source. The other factors that have been included in the checklist for the text fraction include inclusion-exclusion criteria, along with the methods used in the studies [15]. The quality assessment has been conducted with the aim of reducing bias from the study based on the study population, LBP among the participants, measurement procedures, and assessor bindings to the presence of spine pain (yes/no) [16]. The analysis of studies has been conducted via RevMan and Stata where forest and funnel plots were drawn and interpreted [15]. However, the key focus of this meta-analysis and systematic review has been on the statistical data. Still, the thematic analysis has also allowed the researchers to establish a common link between different variables [17].

## 3. Results

### 3.1. Characteristics of Movement

A total of 1887 participants were divided into LBP groups (*n* = 643) and NoLBP groups (*n* = 596). The sample size ranged from 29 to 840.

A meta-analysis was performed for six studies where the angle of lumbar lordosis was compared in people with or even without lower back pain, as shown in Table 2 and Figures 2 and 3. Most studies have reported small insignificant differences amongst groups.

### 3.2. Range of Motion

A meta-analysis of four studies was performed and it was found that there was a consistently reduced movement range in the lumbar spine region with people suffering from lower back pain. A meta-analysis has been performed in Table 3 with the findings listed in Figure 4 with forest and funnel plots. In some of the studies included the groups with chronic or acute lower back pain were compared with other groups showing no back pain signs. Variability was noted in people suffering from lower back pain during flexion. The meta-analysis showed that the flexion in the LBP group was significantly lower (WMD: −0.77; 95% CI: −21.86–2.32; *P* ≤ 0.001, *I*_2_ = 95.2%) than that in the NoLBP group.

Studies which measured bilateral movement were meta-analyzed for extension (Table 4 and Figures 5 and 6), for lateral flexion (Table 5 and Figures 7 and 8), and for rotation (Table 6 and Figures 9 and 10). Meta-analysis showed that the lateral flexion in the LBP group was significantly lower (WMD: −5.58; 95% CI: −10.38 to −0.79; *P*=0.006; *I*_2_ = 75.7%) than that in the NoLBP group. The studies selected were measured for their bilateral movement, that is, in both left and right rotations, and a mean difference was calculated. A significant relationship exists between lower back pain and movement restrictions along with dependent variables that not only efficiently but also effectively cause the same [18].

## 4. Discussion

### 4.1. Analysis of the Current Scenario for Growing of Lumbopelvic Disorder

In most cases, it has been seen that low back pain has contributed to pelvic disorders. The pelvic floor disorder has been noticed to be originating from the displacement of lumbar spines, which hardly has vivid symptoms in most human bodies. However, without or with the symptoms, this disorder reaches an extreme condition to some humans. It has been spotted from many discussions and scientific magazines and journals that the connection between the “low back pain” (LBP) or “spinal pain” and “pelvic floor dysfunction” (PFD) has been evident in the case of women's bodies [19]. The highest number of responses indicated the link between spinal pain and PFD, such as a considerable positive correlation.

### 4.2. Investigation on the Essence of Kinematics

Observing different studies, it has come to light that when the pelvic region muscles are unable to contract, it immediately causes a failure in the urinary tract contraction that results in urinary inconsistency. In the opinion of Aitken et al. [20], adding to it, it has been noticed that the pelvic organ starts prolapsing due to the same reason and gives rise to other abnormalities in the human body. It has been transparent that this phenomenon also disturbs the kinematics of the human body functions and causes PFD.

### 4.3. Analysis of Causes that Develop Further Issues in the Pelvic Region

Low back pain can be derived due to soft-tissue as well as mechanical issues, and these injuries can lead to more pain in their pelvic region. This has been the reason for coming up with more severity, which can lead to more suffering. Furthermore, they have been going through infections, and because of that, they have been facing more casualties.

Due to this reason, more complex problems have been coming up, which can lead to no proper movement of their lives [21]. Hence, it is clear from the discussion that issues developing due to derived spinal pain are related to the pelvic region. This may increase the severity of pain leading to suffering and infections, which might be the reason to other diseases.

### 4.4. Examination of Mitigation Strategies

Here, they should develop proper mitigation strategies at the beginning stage of the pelvic derivation of pelvic. Furthermore, they should easily take physicians' appointments to solve their issues [22]. It is not possible to identify pelvic at their initial stage, but they should pay heed that they should not face any damage so that no issue or further complexity can be generated.

## 5. Conclusion

It can be concluded that lumbopelvic has been derived, so it is too problematic for people to lead their normal lives [23]. There are too many causes behind deriving pelvic disorders such as spinal stenosis, pinched nerves, and herniation. Here, proper analysis of the development of this disorder has been paid heed, and in this regard, it has been identified that spinal pain is the most significant cause [24]. Kinematics has become too vivid a reason for deriving this issue as well, and in this case, all of the explanation has been provided with giving analysis [25]. Possible strategies have been given heed to so that patients can get relieved from this kind of situation to a further extent. Here, for vivid results, primary data has been utilized and the data set given insight into mean and standard deviation values. The analysis of movement in the lumbopelvic region is based on the examination of kinematics such as posture, range of movement like flexion, and extension. This also includes a higher range of movements such as sequential and temporal patterns in case of proprioception, complex functions, physiological movements, or case of complex functions such as walking or lifting. Thus, analysis of all causes for developing various issues in the pelvic region among the patient is very effective, which is generated from spinal pain. It is concluded that people suffering from lower back pain have reduced proprioception and range of movement in the lumbar region when compared to control groups with no lower back pain, which mainly focus on flexion and lateral flexion [26].

Hence, it was concluded from the studies that people with lower back pain have a reduced range and speed of movement, but it is not significant for other characteristics of movement. But people suffering from lower back pain move slowly with low proprioception when compared to control group people. For patients with limited lumbar spine mobility, especially in forward flexion and lateral flexion, early intervention should be performed to reduce pain. For patients who already have low back pain, reducing forward flexion and lateral flexion activities may reduce the pain to a certain extent.

## Figures and Tables

**Figure 1:** PRISMA study over the study methods.

**Figure 2:** Forest plot analysis of lumbar lordosis in the LBP group to NoLBP on lumbar lordosis.

**Figure 3:** Funnel plot analysis of lumbar lordosis in the LBP group to NoLBP on lumbar lordosis.

**Figure 4:** Forest plot analysis of lumbar lordosis in the LBP group to NoLBP on flexion.

**Figure 5:** Forest plot analysis of lumbar lordosis in the LBP group to NoLBP on extension.

**Figure 6:** Funnel plot analysis of lumbar lordosis in the LBP group to NoLBP on extension.

**Figure 7:** Forest plot analysis of lumbar lordosis in the LBP group to NoLBP on the lateral flexion.

**Figure 8:** Funnel plot analysis of lumbar lordosis in the LBP group to NoLBP on the lateral flexion.

**Figure 9:** Forest plot analysis of lumbar lordosis in the LBP group to NoLBP on rotation.

**Figure 10:** Funnel plot analysis of lumbar lordosis in the LBP group to NoLBP on rotation.

**Table 1:** The basic characteristics of the included studies.

Trial	Sample size (LBP/control)	Male/female	Age (*y*), mean ± SD, or range (LBP/control)	Main outcomes	Back pain duration	BMI (LBP/control)
Christie [6]	29 (19/10)	NR	18–46	①	8 years	24.7 ± 3.3/22.8 ± 2.3
Ng [7]	30 (15/15)	30/0	27.9 ± 6.7/27.8 ± 5.9	①④⑤	6.1 years	23.4 ± 1.9/22.7 ± 2.0
Norton [8]	188 (128/60)	85/103	42/39.3	①	7 weeks	NR
Nourbakhsh [9]	840 (420/420)	420/420	20–65	①	6 weeks	25.3/25.6
Youdas [10]	75 (30/45)	75/0	54.9 ± 9/54.8 ± 8.5	①②③	18.7 years	28.9 ± 5.7/26.1 ± 5
Youdas [10]	75 (30/45)	0/75	54.9 ± 8.5/53.4 ± 8.8	①②③	11 years	28.9 ± 5.7/26.1 ± 5
Crosbie [11]	38 (19/19)	13/25	34.0 ± 13.3/28.6 ± 5.4	②④⑤	6 months	24.5 ± 3.6/23.0 ± 2.4
Wong [12]	31 (21/10)	NR	34 ± 10/42 + −8	②③④⑤	1 year	23.6/24.7
Tsai [13]	32 (16/16)	32/0	48.6 ± 7.4/47.9 ± 8.3	③④⑤	2 years	27.9/26.7

NR: not reported; ①: lumbar lordosis; ②: flexion; ③: extension; ④: lateral flexion; ⑤: rotation.

**Table 2:** Comparing the angle of lumbar lordosis in the LBP group to the NoLBP-based group (control).

Study	LBP			Control		
	Mean	SD	Total	Mean	SD	Total
Christie [6]	26.4	9	19	19.3	9.2	10
Ng [7]	26	9	15	25	8	15
Norton [8]	42.5	15.2	128	40.2	14.8	60
Nourbakhsh [9]	37	13	420	38	14	420
Youdas [10]	39	8.1	30	37.5	11	45
Youdas [10]	55.5	10.4	30	52.7	15.3	45

**Table 3:** Flexion-based ROM meta-analysis.

Study	LBP			Control		
	Mean	SD	Total	Mean	SD	Total
Crosbie [11]	48	20	19	50	20	19
Wong [12]	29.8	11.9	20	61.9	9.9	17
Youdas [10] (female)	20.7	8.9	30	23	10.1	45
Youdas [10] (male)	28.6	6.6	30	31	5.7	45

**Table 4:** Extension-based ROM meta-analysis.

Study	LBP			Control		
	Mean	SD	Total	Mean	SD	Total
Tsai [13]	26	7	16	28	8	16
Wong [12]	12.7	5.9	20	15.5	7.4	17
Youdas [10] (female)	56	12	30	56.5	10.4	45
Youdas [10] (male)	42.7	8.8	30	50.1	9.2	45

**Table 5:** The lateral flexion-based ROM meta-analysis.

Study	LBP			Control		
	Mean	SD	Total	Mean	SD	Total
Crosbie [11]	23	11	19	28	13	19
Ng [7]	29.5	5.5	15	31	15	55
Tsai [13]	37	6.5	16	41	6	16
Wong [12]	12.8	4.7	20	23.7	5.4	17

**Table 6:** The rotation-based ROM meta-analysis.

Study	LBP			Control		
	Mean	SD	Total	Mean	SD	Total
Crosbie [11]	12	6	19	12	6	19
Ng [7]	27.5	6.5	15	30.5	10	15
Tsai [13]	43	5	16	47	7	16
Wong [12] (LBP)	9	3.4	20	12.2	4.6	17

## Data Availability

The data used to support this study are available from the corresponding author upon request.
